The article "Optimization Mold and Algorithm of Risk Control for Power Grid Corporations Based on Collaborative Filtering Technology" was published in 2022. Journal: Comput Intell Neurosci.

# Optimization Mold and Algorithm of Risk Control for Power Grid Corporations Based on Collaborative Filtering Technology

**DOI:** 10.1155/2022/3319311

**Published:** 2022-08-01

**Authors:** Longxing Chen, Ping Han

**Affiliations:** The School of Management, Xi'an Jiaotong University, Xi'an 710061, Shaanxi, China

## Abstract

With the ever-changing internal and external environmental factors of enterprises, various uncertainties and risks faced by enterprises are increasing, and the feasibility of financial meltdown is increasing. Research on financial meltdown early warning can help enterprises to prevent the occurrence of peril in advance and take resultful measures to ensure the healthy development of enterprises. If a serious financial meltdown leads to the bankruptcy of enterprises, the financial meltdown is not sudden, but a gradual process. The occurrence of financial meltdown is not only a harbinger, but also predictable. Therefore, it is an urgent question to be solved for listed corporations in China that how to mine the message with early warning function from a large amount of financial data generated in the business process of enterprises. The continuous maturity of data mining technique just solves this question. Based on collaborative filtering technique, this paper analyzes the risk control optimization mold and algorithm of power grid corporations, which is of great signification. After research, this algorithm is 30% better than the traditional algorithm, and it is suitable to be proverbially used.

## 1. Introduction

In the highly competitive market economy, it is not uncommon for listed corporations to get into trouble or even declare bankruptcy due to financial exposures. China's stock market has experienced nearly ten years of development [1]. Faced with the ups and downs of the stock market, some listed corporations have changed from star stocks to junk stocks [2]. Faced with the increasingly complicated economic environment such as increasing competition, tight monetary policy, loss of investor confidence, and fluctuating capital market, whether an enterprise can continue to operate, and how the parties concerned can obtain, message to respond quickly when encountering difficulties are issues of great concern to the enterprise itself, investors, creditors, and even national regulatory agencies and are also a subject worthy of study [3]. The serious financial exposure of the corporation will not only bring huge losses to the production and operation of the enterprise, but also bring huge threats to the relevant stakeholders [4]. It will bring investors' goal of maintaining and increasing the value of properties and even lose money; The bank cannot recover the loan on time; government security regulatory authorities are facing the pressure of disorderly security market [5]. Most foreign studies on this issue regard the enterprise's filing for bankruptcy according to the bankruptcy law as a sign to determine the enterprise's financial distress, that is, define the financial distress as enterprise bankruptcy [6]. Enterprise bankruptcy refers to a kind of litigation procedure carried out according to bankruptcy law when a corporation is insolvent or fails to reach an agreement with creditors outside the court [7]. Taking enterprise bankruptcy as a sign of entering into financial distress, it is easier to determine the research sample because there is a clear demarcation line between bankrupt enterprises and other nonbankrupt enterprises [8]. In fact, the discovery of financial exposures of listed corporations is always a process, and it takes a long time from the incubation period to the outbreak period. In this long time, we can make predictions through certain techniques. In other words, the financial exposure of listed corporations is not sudden, but a process of brewing and development. Listed corporations usually start from a normal financial situation, gradually develop into financial difficulties, and finally fall into financial bankruptcy. Therefore, the occurrence of financial exposures of listed corporations is not only a harbinger, but also completely predictable. Establishing a resultful financial meltdown warning system, judging the corporation's operating status according to the market performance and financial message of listed corporations, and getting the signal of financial deterioration as soon as possible will help relevant stakeholders to make scientific decisions and urge relevant parties to take resultful measures in time to reduce risks and losses [9]. Faced with the increasing harmfulness of financial exposures to listed corporations in China, it is a vital question that most listed corporations in China need to solve how to mine message with early warning function from a large amount of financial data generated in the process of business operation [10]. If we study the bankruptcy behavior of enterprises from the financial aspect, it is obviously inappropriate to confine the questions not only affected by financial factors to the financial domain, and the results will not be satisfactory. Therefore, a better starting point for the study of this question should be to predict whether the corporation's financial situation is healthy, not whether it will go bankrupt [11]. It can be said that the occurrence of financial exposures of any listed corporation is a process of gradual deterioration. It is of great signification that we can find financial exposures in time, reduce losses for relevant investors and creditors, and obtain the greatest benefits, and at the same time enable operators to take resultful measures to improve administration when financial exposures sprout. By analyzing and summarizing the causes of financial exposures of listed corporations and their financial characteristics in different periods, it is of great practical signification for operators, investors, and creditors to protect their own interests, as well as for the security regulatory authorities to monitor the stock market, maintain the fairness of the market, and standardize it [12]. We believe that financial meltdown refers to a kind of financial situation that an enterprise may experience in its production and operation. Due to its poor administration, the enterprise loses its solvency, its financial situation deteriorates, and payment peril occurs. If major strategic adjustments such as reorganization and property injection are not taken, the enterprise will face bankruptcy. Although it seems inevitable that some enterprises will die out in the fierce market competition, the death of enterprises is not a one-off event, but a gradual and continuous accumulation process. According to the famous theory of enterprise life cycle, the development of enterprises can be roughly divided into four stages: budding stage, growing stage, mature stage, and declining stage. When an enterprise enters the declining stage, its products are aging, its technique is outdated, its market is saturated, etc., its competitiveness is weakened, and its profitability and solvency are getting worse and worse. If it fails to make major strategic adjustments in time, it will slowly fall into peril and eventually go bankrupt and liquidate. The continuous maturity of data mining technique and means has just solved this question and opened up a broad space for its financial exposure early warning.

The innovation of this paper lies in the following:

1. Collaborative filtering algorithm is introduced, which is the basis of this article, so we should have a cognition of it. Collaborative filtering technique is the most popular technique in recommendation system, which not only has been deeply improved in academic circles, but also has been well applied in the industry.
2. This paper introduces the collaborative filtering algorithm of k-means clustering, which is the concrete means we adopt in collaborative filtering algorithm. Collaborative filtering based on k-means clustering is to cluster consumers according to k-means clustering algorithm. Its purpose is to separate the target consumers and their clusters from the whole consumer set, and to alleviate the questions of poor scalability and weak implementation performance caused by too large consumer set.
3. The construction of the mold is introduced, so that we can have an overall understanding of the mold. Financial early warning requires that the financial exposures of enterprises can be predicted, so the selected indicators should also be predictive, that is, the possibility of future financial exposures can be predicted by analyzing the historical data formed in the business activities of enterprises, so that the established early warning mold can really predict the financial exposures of enterprises.

This article is divided into five parts:

The first part is the background introduction and the introduction of this article; the second part is the related research of this paper and also mentions this paper. The third part is about the introduction of collaborative filtering. The fourth part is the mold and experimental results, which is the focus of this paper. The fifth part is the conclusion.

## 2. Related Work

Jiang suggested that the artificial neural network analysis means should be introduced to overcome the shortcomings of the traditional economic early warning mold when establishing the bank loan risk early warning system [13]. Armstrong suggested using neural network theory to establish financial early warning mold [14]. Colak suggested a new mold—ZETA mold—to predict the financial failure of enterprises more accurately. By analyzing 53 bankrupt enterprises and 58 nonbankrupt enterprises from 1969 to 1975, the results show that this mold is obviously superior to Z mold in 1968 [15]. Kuo suggested that financial meltdown be defined as “an enterprise going into legal bankruptcy” [16]. Yang and Han suggested that the mold based on option theory should be applied to financial distress early warning research [17]. The multivariable linear discriminant mold suggested by Shih has strict requirements for early warning variables; that is, the early warning variables are required to conform to strict joint normal distribution, but the financial ratio of most enterprises in real economic life cannot meet this requirement [18]. Niu et al. suggested that the financial meltdown should be defined as “a serious liquidation question that cannot be solved unless the operation or structure of an economic entity is restructured on a large scale” [19]. Lu et al. suggested using logistic regression to establish financial early warning mold. The research results show that the scale, financial structure (debt ratio), operating performance (return on properties or working capital ratio), and liquidity (current ratio and quick ratio) of an enterprise are highly correlated with the feasibility of financial exposures [20]. Mansi et al. suggested that the financial meltdown be defined as “an economic phenomenon” in which an enterprise is unable to pay its due debts or expenses, including everything from technological failure of fund administration to bankruptcy and everything in between [21]. Galvez et al. suggested that the neural network system should be used to resultfully predict the bankruptcy of the corporation with an accuracy of up to 97% [22].

Early warning analysis of listed corporations' financial situation not only is the focus of attention of people from all walks of life, but also has vital guiding signification for the future development of listed corporations. Data mining can process the business message of the enterprise, process the data quickly and efficiently, find out the deterioration of the financial targets, and judge the different stages of the financial meltdown that the enterprise is in. Based on collaborative filtering technique, this paper studies the risk control optimization mold and algorithm of power grid corporations, which is of great signification.

## 3. Collaborative Filtering Technique

### 3.1. Collaborative Filtering and Recommendation

With the advent of the age of big data and Internet, it has become an inevitable trend for people to enter the age of message overload. The scale of global data has increased from the original level to the current level. Compared with the structured data, which is easy to store in the past, the proportion of unstructured data such as audio, video, pictures, and geographical location message has gradually increased, reaching about 80%. Internet has its own unique characteristics and advantages. First of all, it can realize complete resource sharing; secondly, it is possible to realize efficient and convenient communication through the Internet; third, the development of Internet technique has achieved better fairness. The rapid growth of message on the Internet, on the one hand, makes people's access to more and more message resources, which brings great convenience to people. On the other hand, people are often confused when faced with a huge amount of message resources, and they have to spend more time and energy searching for helpful message. The phenomenon of “message overload” is becoming more and more serious. Information overload is not only a unique question of the Internet, but also a similar phenomenon in real life, compared with the limited amount of message that the human brain can handle at the same time. That is to say, how to improve the message retrieval efficiency in the complicated message has become a research hotspot. The appearance of recommendation system just solves the question of data redundancy caused by long data. On the one hand, from the consumer's point of view, it can avoid the waste of time and energy caused by searching for complicated data, and improve the consumer's Internet experience; on the other hand, Internet service providers can accurately recommend the content they want to promote and recommend to consumers, thus realizing low-cost and high-return investment.

Whether the consumer message is obtained by explicit tracking or implicit tracking, it can be represented by a consumer-item scoring matrix *R*. *R* is a *m* × *n*-order matrix, where *m* represents the number of consumers and *n* represents the number of items. For displaying tracking preference message, each element *Rij* in the matrix represents the *i* th consumer's rating value for the *j* th item, its possible values are *Z*={*v*,…, *V*} ∪ {•}, *v* is the minimum rating value (usually 1), *V* is the maximum rating value (usually 5 or 7), and • indicates that the consumer has not rated the item as shown in Table 1.

Let the similarity sim(*u*_*a*_, *u*_*i*_) among the consumers in the nearest neighbor sets *U*_*n*_={*u*_1_, *u*_2_,…, *u*_*k*_}, *u*_*a*_ ∉ *U*_*n*_, *U*_*n*_, and *u*_*i*_(1 ≤ *i* ≤ *k*) of the consumer group *u*_0_ with higher similarity be arranged in descending order.

Person correlation coefficient is

(1) $$\begin{array}{c} \text{sim}\left(u,v\right)=\frac{\Sigma_{i\in I_{uv}}\left(R_{u,i}-{\bar{R}}_{u}\right)\left(R_{v,i}-{\bar{R}}_{v}\right)}{\sqrt{\Sigma_{i\in I_{uv}}{\left(R_{u,i}-{\bar{R}}_{u}\right)}^{2}}\sqrt{{\sum_{i\in I_{uv}}\left(R_{v,i}-{\bar{R}}_{v}\right)}^{2}}}, \end{array}$$

where *u* and *v* represent two consumers in the consumer space; sim(*u*, *v*) indicates the similarity between *u* and *v*; *I*_*uv*_ indicates the common score item set of *u* and *v*, namely, *I*_*uv*_={*i* ∈ *I|r*_*u*,*i*_ ≠ •∧*r*_*v*,*i*_ ≠ •}; *R*_*u*,*i*_ and *R*_*v*,*i*_, respectively, indicate the ratings of *u* and *v* for item *i*; and ${\bar{R}}_{u}\text{ and }{\bar{R}}_{v}$ indicate the average rating of all items in *u* and *v*, respectively.

Let *u* and *v* represent the scoring vectors of consumers *u* and *v*, respectively, then the similarity between *u* and *v* is

(2) $$\begin{array}{c} \text{sim}\left(u,v\right)=\cos\left(u,v\right)=\frac{\Sigma_{i\in I_{uv}}R_{u,i}R_{v,i}}{\sqrt{\Sigma_{i\in I_{uv}}R_{u,i}{}^{2}}\sqrt{\Sigma_{i\in I_{uv}}R_{v,i}{}^{2}}}. \end{array}$$

The similarity between consumers *u* and *v* is calculated by the following formula:

(3) $$\begin{array}{c} \text{sim}\left(u,v\right)=1-\frac{\Sigma_{i\in I_{uv}}{\left(N_{u,i}-N_{v,i}\right)}^{2}}{\left|I_{uv}\right|}. \end{array}$$

Personalized recommendation system is an intelligent recommendation system for big data, which can make corresponding personalized decision support for customers of e-commerce platform. Due to the efficient decision-making mechanism and good recommendation performance, personalized recommendation system has been proverbially used in various platforms. Recommendation system is a resultful solution to the question of message overload. According to the characteristics of consumers, it recommends the targets that meet the needs of consumers and realizes personalized service. The fundamental reason why recommendation system can provide consumers with interesting message is that it relies on consumers' historical behaviors to analyze consumers' needs. Simply put, the essence of recommendation is to link external message through certain ways and means. Among them, collaborative filtering technique is the most popular technique in recommendation system, which has been deeply improved in academic circles and well applied in the industry. The most fundamental idea of synergetic coincidence algorithm is to collaborate among consumers, that is, to make recommendations based on the data of consumers with the same attributes or similarities, which will greatly increase the density of data and the credibility of recommended data. By improving these two aspects, the questions of data sparsity and low credibility are solved, thus improving the accuracy of recommendations.

### 3.2. Collaborative Filtering Algorithm Based on *k*-Means Clustering

Collaborative filtering algorithm to resultfully alleviate data sparsity and improve recommendation accuracy belongs to collaborative filtering algorithm based on memory. In order to find the neighbor set similar to the target consumer, we need to traverse all consumers in the system. However, with the continuous expansion of the system scale, new consumers and projects will continue to join, and the shortcomings of the system, such as poor scalability, are becoming more and more serious. To alleviate this situation, many scholars put forward collaborative filtering based on mold. The difference between collaborative filtering based on k-means clustering and general collaborative filtering based on consumers lies in the step of mining neighboring consumers. No matter what kind of mold is based on, the common point of the algorithms is to use historical data to train the mold, and the training of the mold is basically done offline. Compared with the collaborative filtering based on memory, the collaborative filtering algorithm based on mold can resultfully alleviate the shortcomings of the former algorithm. Especially, the advantages of clustering technique, such as strong usability and good scalability for large-scale data sets, can resultfully overcome the above disadvantages. So now we will study the collaborative filtering of k-means clustering. Collaborative filtering based on k-means clustering is to cluster consumers according to k-means clustering algorithm. Its purpose is to separate the target consumers and their clusters from the whole consumer set, and to alleviate the questions of poor scalability and weak implementation performance caused by too large consumer set. Clustering analysis is an exploratory analysis, which is a process of dividing chaotic data into different classes or clusters by certain standards. It is based on the idea of “birds of a feather flock together.” Through certain attributes such as Pearson distance, the similarity of targets within a class and the dissimilarity of targets between classes are as large as possible. Finally, through the clustering results, we can find some connection between data attributes.

The following is a detailed description of the algorithm:

  Step 1 : Determine *k* initial centroids from the set *M*, and set them as *Ss*_1_, *Ss*_2_,…, *Ss*_*N*_, where centroids can be randomly selected.
  Step 2 Calculate the distance *d* between the noncentroid point and each centroid point. The distance can be measured by Euclidean distance, as shown below:
  (4) $$\begin{array}{c} d\left(x,y\right)=\sqrt{{\left(x_{1}-y_{1}\right)}^{2}+{\left(x_{2}-y_{2}\right)}^{2}+\ldots {\left(x_{n}-y_{n}\right)}^{2}}=\sqrt{\sum_{i=1}^{n}{\left(x_{i}-y_{n}\right)}^{2}}. \end{array}$$
  Step 3 Assign the noncentroid point to the set corresponding to the nearest centroid point and set it to *Sn*_1_, *Sn*_2_ … *Sn*_*N*_.
  Step 4 Repeat steps 2 and 3.
  Step 5 Until the centroid does not change or the iteration stop condition is reached, the final clustering result is given, and the algorithm ends.

Clustering algorithm is proverbially used in many domains, such as recommendation system, deep learning, and intelligent computing. The collaborative filtering algorithm based on k-means clustering first divides consumers into K clusters through consumer message, which directly reduces the data base compared with the general collaborative filtering algorithm based on consumers. At the same time, after mining the neighbor consumers, only the results of the first K nearest neighbors (*K* is far less than the total number of consumers *N*) are adopted, which reduces the time complexity of the algorithm to some extent. We can intuitively feel the improvement of operation efficiency in the experiment. The advantage of introducing clustering algorithm into recommendation lies in that the search of target consumers can only be carried out in the cluster containing the target consumers, instead of searching in the whole database. Therefore, the recommendation speed can be improved. This algorithm can reduce the consumer base by clustering consumers, thus improving the efficiency of recommendation to a certain extent. Its simple mold is universal, and it shows good scalability on large-scale data sets.

## 4. Model Establishment and Experimental Results

At present, domestic and foreign researches are mostly devoted to screening financial ratios or variable combinations that are both explanatory and stable to build molds. Statistical data mining technique plays a vital role in establishing financial meltdown early warning mold, and the early financial meltdown early warning molds are all based on statistical technique. Discriminant analysis is a statistical analysis means that discriminates the categories of research targets. Discriminant analysis must know the classification of the observed targets and some variable values indicating the characteristics of the observed targets. Discriminant analysis is to screen out variables that can provide more message and establish discriminant function, so that the misjudgment rate of the deduced discriminant function when classifying observation samples is minimal. The structure of data mining system is shown in Figure 1.

From previous empirical studies, it can be seen that most researchers are committed to screening financial ratios or variable combinations that are both explanatory and stable to build molds. Although researchers are trying to prove that the variables they use are superior to other research results, there is no consistent conclusion at present, even a consistent means of screening variables. The design of financial early warning index system should be able to fully reflect the financial status of listed corporations in terms of profitability, growth ability, debt paying ability, property administration ability, and cash flow, so as to analyze the capabilities of enterprises in all aspects, so as to reveal and judge the financial status and future development trend of enterprises as comprehensively as possible. Discriminant financial meltdown early warning mold aims to study the classification of two types of corporations. One is financial meltdown corporation, and the other is financial health corporation. Based on this, a discriminant function is established to discriminate and classify any corporation, borrower, and security issuer. The steps of building a financial early warning system are shown in Figure 2.

In order to expand the business scale or meet the needs of business turnover, almost every listed corporation is in debt, but the debt ratio is different. High debt ratio usually becomes risky business, while low debt ratio may fall into the stereotype of conservative business. As there are many indicators of financial exposure warning, it is impossible to include all financial targets in the study. If too many indicators are selected, the resultfulness and practicability of the mold will be affected. The univariate analysis compares the corporation's vital financial ratios with the standards of the same industry to see if there is a big difference between them, and observes the trend of financial ratios to predict the financial meltdown. Regardless of the level of debt, it is the basic premise for listed corporations to repay their debts when they are due. If a listed corporation fails to repay its due debts, it may be taken over by creditors or judged bankrupt by the court. Therefore, the financial targets related to solvency are often used as vital indicators to examine the financial exposures of listed corporations.

Suppose *Y* is used to record the financial status of listed corporations, the financial meltdown occurs, and it is recorded as *Y*=1; if the financial meltdown does not happen, it will be recorded as *Y*=0. *Y* depends on another unobservable variable *V*, while *V* has a certain functional relationship *V*=*f*(*X*) with the predicted variable *X* we use, which is assumed to be linear for simple design:

(5) v=βx+iεi.

The value of *V* determines whether the event *Y* occurs, assuming that when *Y*=1 is equivalent to *V* > 0, then *Y*=0 is equivalent to *V* ≤ 0. Therefore, the feasibility of the event (*Y*=1) occurring is

(6) $$\begin{array}{c} P\left(Y=1\right)=P\left(V>0\right)=P\left(\varepsilon_{i}>-\beta x_{i}\right). \end{array}$$

In order to estimate formula *v*=*βx*_*i*_+*ε*_*i*_ according to a certain sample, it is necessary to select a certain feasibility distribution function for *ε*_*i*_. The feasibility distribution function of *ε*_*i*_ is *F*(*t*), and the feasibility distribution function is

(7) $$\begin{array}{c} F\left(t\right)=\frac{e^{1}}{1+e^{1}}. \end{array}$$

From *F*(−*t*)=1 − *F*(*t*), formula *P*(*Y*=1)=*P*(*V* > 0)=*P*(*ε*_*i*_ > −*βx*_*i*_) can be transformed as follows:

(8) $$\begin{array}{c} P\left(Y=1\right)=\frac{e^{\beta x_{i}}}{1+e^{\beta x_{i}}}. \end{array}$$

When the *i* th sample is a financial meltdown corporation, *Y*_*i*_=1. When the *i* rd sample point is a nonfinancial meltdown corporation, *Y*_*i*_=0.

*X*_*i*_=(*Xi*1, *Xi*2,…, *Xik*) is the index variable of the *i* nd sample point:

(9) $$\begin{array}{c} \beta x_{i}=\beta_{0}+\beta_{1}x_{i1}+\beta_{2}x_{i2}+\ldots +\beta_{k}x_{ik}. \end{array}$$

From *P*(*Y*=1)=*e*^*βx*_*i*_^/1+*e*^*βx*_*i*_^, you can get

(10) $$\begin{array}{c} \ln\frac{p}{1-p}=\beta x_{i}=\beta_{0}+\beta_{1}x_{i1}+\beta_{2}x_{i2}+\ldots +\beta_{k}x_{ik}. \end{array}$$

The selected financial exposure warning indicators should be able to be obtained by calculating the financial data of listed corporations; that is to say, the selected indicators should not only meet the purpose of financial exposure warning, but also be supported by data, and the message required for each data indicator must be easily available. Otherwise, the selected financial meltdown early warning indicators will lose any practical signification because there is no way to calculate them. A failed enterprise has less cash but more accounts receivable. When the cash and accounts receivable are added together and included in liquid properties or current properties, the difference between a failed enterprise and a successful enterprise will be covered up. It is the premise of the existence and development of listed corporations, and the basic condition for listed corporations to survive in the market is to make ends meet. From the market point of view, a long-term loss-making listed corporation always withdraws from the market when it exhausts all its resources. Investors, creditors, managers of listed corporations, and even government managers are increasingly paying attention to the profitability of listed corporations. As shown in Figures 3–5, the mold-based collaborative filtering algorithm used in this algorithm is superior to the traditional content-based collaborative filtering algorithm. With the increase of game times and time, the feasibility of fraud by message providers gradually converges.

Financial early warning requires that the financial exposures of enterprises can be predicted, so the selected indicators should also be predictive; that is, the possibility of future financial exposures can be predicted by analyzing the historical data formed in the business activities of enterprises, so that the established early warning mold can really predict the financial exposures of enterprises. Taking total liabilities as the base is to consider the transformation relationship between long-term liabilities and current liabilities. However, the total liabilities only consider the scale of liabilities, but not the liquidity of liabilities, that is, the debt structure of enterprises. Therefore, there is a great misjudgment for some enterprises that are in peril due to short-term solvency. The index of “total properties” does not take into account the components of properties, and different property items play different roles in the business process, which is not conducive to predicting the profitability of enterprise properties. Asset administration ability is used to measure the efficiency of listed corporations in property administration. The profitability of listed corporations is the result, while the property administration ability is the cause. Listed corporations with good performance should have good property administration ability. Therefore, the financial targets reflecting the property administration ability are also vital indicators used to examine the financial exposures of listed corporations. As can be seen from Tables 2–4, Figures 6–8, the algorithm in this article is 30% better than the traditional algorithm, and it is suitable for being proverbially used. When the consumer moves to the right, it can be kept at a highly stable level.

The selected early warning indicators can sensitively reflect the changes of enterprise operation activities; that is, once the risk factors occur, they can be quickly reflected in the indicator values. Multivariate mold is a multivariate function formula established by using the idea of multivariate mold; that is, a variety of financial targets of an enterprise are weighted and aggregated to generate the total discriminant score of the enterprise to predict the possibility of financial meltdown. Multivariate mold can be regarded as an extension of univariate mold; that is, different financial targets are integrated into one mold. The construction of enterprise financial exposure early warning index system should be scientifically designed according to the causes of enterprise financial exposures, and the index system should be able to make a scientific description of each cause. Profitability is the ability of capital appreciation of enterprises, which is the premise of the existence and development of listed corporations and the comprehensive embodiment of financial structure and operating performance. If an enterprise's profitability is stable, it will have enough surplus to face various possible financial exposures, and the possibility of financial meltdown will be lower. Therefore, the financial targets related to the profitability of listed corporations are also used as vital indicators to establish financial exposure early warning molds.

## 5. Conclusions

The essence of financial distress is the concentrated outbreak of large-scale and high-intensity financial exposures, which is mainly manifested in the extreme deterioration of financial situation, payment peril, and even bankruptcy. Generally speaking, the financial data of listed corporations in China can predict the feasibility of financial exposures in the future; that is to say, the financial targets of listed corporations in China contain certain message content, and consumers of financial data can accurately predict whether financial exposures will occur in the future according to the message provided by the balance sheet, profit statement, and cash flow statement of listed corporations. From the financial point of view, financial distress refers to an enterprise's loss of solvency, that is, its inability to repay its due debts, such as bankruptcy, default on preferred stock dividends, and inability to repay debts. The application of mold-based collaborative filtering technique to financial message processing and financial meltdown early warning has greatly improved the accuracy of financial meltdown early warning, eliminated many external interference factors, and made more hidden message in financial data appear. After research, this algorithm is 30% better than the traditional algorithm, and it is suitable to be proverbially used.

## Figures and Tables

**Figure 1:** Structure of data mining system.

**Figure 2:** Steps to build a financial early warning system.

**Figure 3:** Change of equilibrium point.

**Figure 4:** Game process.

**Figure 5:** Game equilibrium point change.

**Figure 6:** Income comparison.

**Figure 7:** Response comparison.

**Figure 8:** Lifting diagram.

**Table 1:** User-project rating matrix.

	*i*_1_	…	*i*_*j*_	…	*i*_*n*_
*u*_1_	*R*_1,1_	…	*R*_1,*j*_	…	*R*_1,*n*_
…	…	…	…	…	…
*u*_*i*_	*R*_*i*,1_	…	*R*_*i*,*j*_	…	*R*_*i*,*n*_
…	…	…	…	…	…
*u*_*m*_	*R*_*m*,1_	…	*R*_*m*,*j*_	…	*R*_*m*,*n*_

**Table 2:** Income comparison.

	0	10	20	30	40	50	60	70	80	90	100
Algorithm	56	55	42	39	46	45	51	57	59	60	62
Traditional algorithm	49	50	43	51	53	41	37	52	50	46	55

**Table 3:** Response comparison.

	0	10	20	30	40	50	60	70	80	90	100
Algorithm	66	59	60	41	57	55	62	67	61	70	72
Traditional algorithm	57	55	62	49	44	51	53	44	60	54	56

**Table 4:** Lifting diagram.

	0	10	20	30	40	50	60	70	80	90	100
Algorithm	3.7	2.5	3.1	3.5	1.9	2.6	3.3	3.6	2.7	2.5	3.4
Traditional algorithm	2.9	3	3.4	2.5	2.6	1.8	2.4	3.3	1.9	2.4	3.1

## Data Availability

The data set can be accessed upon request.
